# Efficacy of Imiquimod-Based Transcutaneous Immunization Using a Nano-Dispersed Emulsion Gel Formulation

**DOI:** 10.1371/journal.pone.0102664

**Published:** 2014-07-15

**Authors:** Pamela Stein, Karsten Gogoll, Stefan Tenzer, Hansjörg Schild, Stefan Stevanovic, Peter Langguth, Markus P. Radsak

**Affiliations:** 1 Institute for Immunology, Johannes Gutenberg-University Medical Center, Mainz, Germany; 2 Biopharmaceutics and Pharmaceutical Technology, Johannes Gutenberg-University, Mainz, Germany; 3 Department of Immunology, Eberhard Karls-University Tübingen, Tübingen, Germany; 4 Third Department of Medicine, Johannes Gutenberg-University Medical Center, Mainz, Germany; Mie University Graduate School of Medicine, Japan

## Abstract

**Background:**

Transcutaneous immunization (TCI) approaches utilize skin associated lymphatic tissues to elicit specific immune responses. In this context, the imidazoquinoline derivative imiquimod formulated in Aldara applied onto intact skin together with a cytotoxic T lymphocyte (CTL) epitope induces potent CTL responses. However, the feasibility and efficacy of the commercial imiquimod formulation Aldara is limited by its physicochemical properties as well as its immunogenicity.

**Methodology/Principal Findings:**

To overcome these obstacles, we developed an imiquimod-containing emulsion gel (IMI-Gel) and characterized it in comparison to Aldara for rheological properties and *in vitro* mouse skin permeation in a Franz diffusion cell system. Imiquimod was readily released from Aldara, while IMI-Gel showed markedly decreased drug release. Nevertheless, comparing vaccination potency of Aldara or IMI-Gel-based TCI in C57BL/6 mice against the model cytotoxic T-lymphocyte epitope SIINFEKL, we found that IMI-Gel was equally effective in terms of the frequency of peptide-specific T-cells and *in vivo* cytolytic activity. Importantly, transcutaneous delivery of IMI-Gel for vaccination was clearly superior to the subcutaneous or oral route of administration. Finally, IMI-Gel based TCI was at least equally effective compared to Aldara-based TCI in rejection of established SIINFEKL-expressing E.G7 tumors in a therapeutic setup indicated by enhanced tumor rejection and survival.

**Conclusion/Significance:**

In summary, we developed a novel imiquimod formulation with feasible pharmaceutical properties and immunological efficacy that fosters the rational design of a next generation transcutaneous vaccination platform suitable for the treatment of cancer or persistent virus infections.

## Introduction

Transcutaneous immunization (TCI) approaches are increasingly gaining interest by vaccine developers since they incorporate all desirable properties of an ideal cancer vaccine, in terms of defined antigen specificities, targeting of specific APC populations and well-defined adjuvants [1], [2]. Besides the advantage of patient self-medication, such easy-to-use vaccines lack the need for injections. In particular, needle-borne accidents in both medical personnel and patients will be circumvented. This is a priority issue conceded by the WHO based on the medical and socioeconomic consequences of needle injuries [3], [4]. From an immunological point of view the skin is an attractive target for shaping immune responses: the delivery of antigens is controlled and specifically targeted to skin resident APC [5] in direct conjunction with an adjuvant eliciting potent adaptive immune responses as pioneered by Glenn and coworkers [6]. While parenteral (subcutaneous or intramuscular) vaccine delivery systems are not as well controlled in terms of drug release and targeting of specific immune organs, the drug dosage and targeting to the skin in transcutaneous approaches can be more easily and specifically achieved, e. g. by specific modifications of the vaccine as recently demonstrated for a nanoparticle-formulated DNA vaccine [7].

We have previously shown that the concurrent administration of a cytotoxic T lymphocyte (CTL) epitope together with the TLR7 agonist imiquimod onto intact skin elicits potent primary CTL responses [8]. While imiquimod-based TCI has been successfully applied to experimental rodent models by us and others [5], [9]–[11], the clinical efficacy of topical imiquimod in patients with HPV infections [12] or skin cancers [13] makes it very likely that novel imiquimod-based vaccination concepts may also be effective in humans. This assumption is further supported by the finding that imiquimod efficiently enhances T-cell responses when used as an adjuvant in humans in pilot studies with melanoma patients immunized against NY-ESO-1 protein [14] or patients with prostate cancer treated with a multi peptide vaccine [15].

CTL responses induced by TCI with imiquimod based on the commercial formulation in Aldara rapidly fade away, resulting in poor memory formation and only partial tumor protection [5], [9]. However, T-cell responses and tumor protection can be rescued by additional stimuli, e.g. by CD40 ligation [5], [9] or low dose UV-B irradiation [5]. This highlights the importance of “high-quality” T cell responses that confer effective memory responses to achieve anti-tumor immunity and furthermore suggests that imiquimod formulated in Aldara is not an ideal preparation for TCI purposes. We have also recently shown that various imiquimod formulations considerably differ in their release of imiquimod and their potency to induce CTL responses in TCI [16].

Based on this, we hypothesized that for effective TCI it is not necessary for imiquimod to be solubilized e. g. in isostearic acid, which is responsible for Aldara-induced TLR7-independent adverse skin reactions [17]. We therefore generated an imiquimod-containing emulsion gel (IMI-Gel) in which the crystalline imiquimod is nano-dispersed in a hydrophilic polyacrylate gel containing a lipophilic dispersed phase. We compared IMI-Gel to Aldara in terms of drug permeation across mouse skin. Not surprisingly, imiquimod release over time occurred significantly faster from Aldara compared to IMI-Gel. However, when IMI-Gel was compared to Aldara-based TCI, both imiquimod formulations showed equal potency in the induction of primary CTL responses. More importantly, IMI-Gel was also at least as effective as Aldara induced TCI in a therapeutic tumor vaccination model, indicating the induction of high quality memory T cell responses. Collectively, these results support the notion that Aldara is not an ideal formulation for vaccination purposes and that the development of revised preparations and a deeper understanding of the underlying mechanisms may harbour the key for the rational design of a next-generation TCI platform that can be used for the treatment of cancer.

## Results

### Physicochemical properties of imiquimod formulation IMI-Gel

Based on our previous finding that despite the presence of crystalline imiquimod various imiquimod formulations can induce CTL responses in TCI [16] we hypothesized that solubilisation of imiquimod is not required for successful TCI. We therefore manufactured a hydrophilic polyacrylate gel in which imiquimod is nano-dispersed in a lipophilic phase (IMI-Gel). Imiquimod crystals were dispersed within the gel formulation (Fig. 1A) and had an average mean size of 335 nm±79 nm post manufacturing. Martin diameter of imiquimod crystals ranges from approximately 100 nm–500 nm. The particle size remained stable after 9 months of storage at room temperature (286 nm±12 nm calculated as average mean of three DLS z-average values), excluding potential Ostwald ripening processes (Fig. 1B), and there was no phase separation during the storage period. In summary, this indicates an accurate stability of the IMI-Gel formulation.

**Figure 1:** In vitro characterization of IMI-Gel. To characterize IMI-Gel and Aldara, imiquimod containing formulations were analyzed in terms of **A)** presence of imiquimod crystals in IMI-Gel using electron microscopy, **B)** sizes (mean+SD) of imiquimod-particles in IMI-Gel immediately or 9 months after manufacturing (under room conditions) and **C)** flow curves defining rheological characteristics.

As shown in Fig. 1C, rheologic measurements demonstrated a thin fluid consistency of Aldara, similar to common dermally applied lotions. In contrast, for IMI-Gel we detected a high viscosity resulting in an approx. 20-fold increased shear stress at comparable shear rates. Taken together, imiquimod formulated in IMI-Gel was pharmaceutically different compared to Aldara, but was stable with acceptable pharmaceutical quality properties and therefore suitable for further functional evaluation.

### Imiquimod formulated in IMI-Gel shows lower permeation through murine skin compared to Aldara

TCI approaches offer the advantage of gaining direct access to skin-resident DC and therefore facilitate their stimulation, migration and subsequent antigen presentation in draining lymph nodes. To this end, imiquimod as the active component or adjuvant in our TCI approach should be targeted to the skin and remain there for optimal DC activation. To address this, we explored the skin permeation of both imiquimod formulations and placed skin samples in a Franz-diffusion-cell system (Fig. 2A), either applying Aldara or IMI-Gel on isolated mouse skin. Subsequently, we analyzed the concentration of imiquimod in the acceptor medium over time. As depicted in Fig. 2B, 11.5% of imiquimod was released by Aldara (grey line), while only 1% imiquimod permeated across the skin when formulated in IMI-Gel (black line). To determine the amount of imiquimod within the skin, we treated mice either with IMI-Gel or Aldara on an area of 6 cm^2^ on the shaved backs. After 3 hours, the amounts of the respective formulations remaining on the skin were harvested using gauze. Afterwards 1 cm^2^ of skin was prepared and fat was carefully removed. Samples were collected in extraction buffer and then hackled with an ultra turrax. The amount of imiquimod found in the supernatant of centrifuged gauze or skin samples was analyzed by HPLC. As shown in Fig. 2C (left panel) 40% of imiquimod applied with IMI-Gel remained on the skin surface 3 hours after treatment, whereas 19% were recovered after Aldara treatment (statistically not significant). Analyzing the amount of imiquimod within the skin (Fig. 2C right panel) revealed that slightly more imiquimod was found in the skin of IMI-Gel treated (14 µg/cm^2^±3 µg/cm^2^) compared to Aldara treated (11 µg/cm^2^±1.7 µg/cm^2^) mice (statistically not significant).

**Figure 2:** Imiquimod passes mouse skin *in vitro* more rapidly when formulated in Aldara than in IMI-Gel. **A)** Release of imiquimod as the active component was detected with a modified Franz-diffusion-cell model. **B)** Shaved skin of C57BL/6 mice (n = 6) was ablated and afterwards treated with Aldara or IMI-Gel (each 50 mg). The imiquimod concentration in the acceptor medium was determined after various time points as indicated using HPLC (UV absorption 245 nm). *Significant difference with p<0.05 by Wilcoxon signed rank test. **C)** C57BL/6 mice (n = 3) were with Aldara or IMI-Gel (each 50 mg/6 cm^2^) on. After 3 hours mice were sacrificed and remaining formulation was removed with gauze. 1 cm^2^ of treated skin was prepared, fat removed and subsequently hackled with an ultra turrax. The amount of imiquimod recovered from the skin surface (left panel) and within the skin (right panel) was determined using HPLC.

These results indicate that imiquimod formulated in Aldara was taken up across the skin more effectively allowing systemic exposure of the drug, while imiquimod formulated in IMI-Gel appeared to remain in and on top of the skin.

### IMI-Gel and Aldara are equally potent in inducing peptide specific CTL responses

So far, our results indicated a lower drug permeation of imiquimod when formulated in IMI-Gel. We asked whether or not this is of relevance for TCI efficacy since imiquimod should specifically activate skin DCs [5], [10], [18]. Therefore, a lower skin permeation of IMI-Gel imiquimod may not necessarily be a disadvantage for TCI induced immune responses. To directly address this, we compared the potency of IMI-Gel or Aldara treatment regarding the induction of peptide-specific CTL responses. This was done either by administering Aldara together with the major histocompatibility complex (MHC) class-I-restricted T cell epitope OVA_257–264_ (SIINFEKL, SIIN) or IMI-Gel followed by the additional treatment with OVA_257–264_ in officinal cremor basalis on two consecutive days on the dorsal region of C57BL/6 mice. Analyzing the frequency of peptide-specific T cells via MHC I tetramer stainings of blood samples revealed comparable amounts in both immunized groups (Fig. 3A). We then determined the lytic capacity of cytotoxic T cells with an *in vivo* cytotoxicity assay (Fig. 3B) and found that the majority of target cells (75%) was specifically lyzed after Aldara-induced TCI, as described previously [5], [9]. Interestingly, the CTL response induced by TCI with IMI-Gel was comparable and indistinguishable from the Aldara-induced response despite a >10 fold less drug permeation across mouse skin. These results suggest that it is important for CTL induction in imiquimod-based TCI that the drug is targeted to the skin and that it does not need to be delivered systemically.

**Figure 3:** IMI-Gel and Aldara are equally potent in inducing primary CTL-responses. C57BL/6 mice were shaved on their backs and afterwards immunized on two consecutive days with either Aldara (50 mg) together with SIINFEKL (100 µg) or IMI-Gel (50 mg) and officinal cremor basalis together with SIINFEKL or left untreated (untreated control). **A)** The frequency of peptide-specific CD8^+^ T cells in the blood (mean and SD) and **B)** *in vivo* cytolytic activity 24 hours (mean and SD) after transfer of peptide-loaded target cells was assessed. Depicted are the cumulative results of two independent experiments with n = 6 for the tetramer staining and three independent experiments with n = 9 for the cytotoxicity assay. *Significant difference with p<0.05 by one-way ANOVA with Bonferroni’s posttest.

### Transcutaneous delivery of imiquimod induces superior CTL responses compared to s. c. or oral application

In case it is indeed important for imiquimod-based TCI that the drug remains locally within the skin, then an imiquimod-based vaccination would be less effective if the skin was passed by via s. c. injection. To clarify this, we vaccinated mice as before with IMI-Gel-based TCI. As important controls and to exclude the induction of CTL responses was due to skin irritations by the shaving procedure or independent of the CTL epitope, we included a group treated with IMI-Gel without the CTL epitope SIINFEKL or a group treated with the SIINFEKL (in officinal cremor basalis) without IMI-Gel. For comparison, we added low amounts of sterile water to IMI-Gel and the CTL epitope to allow aspiration in a syringe and injected this s. c. in the dorsal neck region. As depicted in Fig. 4, the IMI-Gel s. c. administration did neither induce specific T cells nor specific cytotoxicity. Also, the treatments with IMI-Gel or the CTL epitope alone were unable to elicit CTL responses. To furthermore exclude the possibility that IMI-Gel is orally taken up, e. g. by grooming post topical application on the back, we performed additional experiments where a group of mice was fed with IMI-Gel and peptide using an oral gavage on two consecutive days. As shown in Fig. 4, the oral delivery of IMI-Gel did not elicit a CTL response. In contrast, IMI-Gel-based TCI was again effective in terms of frequency of specific CTL and cytolytic activity. Importantly, we used the identical pharmaceutically active components (IMI-Gel and peptide) at the same doses.

**Figure 4:** The route of IMI-Gel application influences vaccination efficacy. C57BL/6 mice were shaved on their backs and received the following treatments: untreated (untreated control), IMI-Gel with SIINFEKL (100 µg) (IMI-Gel TCI) on two consecutive days, IMI-Gel alone (IMI-Gel without SIIN) on two consecutive days, oral IMI-Gel (50 mg) with SIINFEKL (100 µg) on two consecutive days (IMI-Gel p. o.) or s. c. once with IMI-Gel (100 mg) diluted with SIINFEKL (200 µg) and distilled water into the neck. **A)** The frequency of peptide-specific CD8^+^ T cells in the blood (mean and SD) and **B)** *in vivo* cytolytic activity 24 hours (mean and SD) after transfer of peptide-loaded target cells was assessed. Depicted are the cumulative results of two independent experiments with n = 7 for IMI-Gel treated groups and n = 4 for controls. *Significant difference with p<0.05 by Students *t* test.

These results clearly show that the transcutaneous delivery of imiquimod is important for vaccine efficacy and superior to the parenteral route of application.

### IMI-Gel induced TCI increases tumor protection in a therapeutic model

After having demonstrated comparable primary immune responses via Aldara or IMI-Gel-based TCI (Fig. 3), we wanted to evaluate the potency of both imiquimod formulations regarding the induction of high-quality memory CTL responses as required for tumor protection. We therefore tested both TCI treatments in a therapeutic tumor model, in which mice were inoculated s. c. with E.G7 thymoma cells, expressing ovalbumin as a surrogate tumor antigen. After the tumors became palpable, mice were left untreated or vaccinated as described before in weekly intervals over a period of three weeks. Unimmunized control mice showed a durable tumor growth in 12 of 17 animals (Fig. 5A). In the five animals with spontaneous tumor rejection, we detected up to 2% peptide-specific CTL (data not shown), indicating potential endogenous immunogenicity of the E.G7 tumor cells. Importantly, in the 12 animals with growing solid tumors no specific CTL responses were detectable and the mice had to be sacrificed in the end (overall survival 29.4%; median survival 25 days).

**Figure 5:** Delayed tumor growth and tumor protection after IMI-Gel application. E.G7 thymoma cells (4×10^5^ s.c.), expressing SIINFEKL, were injected into the flank of C57BL/6 mice. After the tumor was palpable mice were immunized as indicated on two consecutive days in weekly intervals over a period of three weeks or left untreated. **A)** The tumor size and **B)** the survival were monitored. Depicted are the cumulative results of three independent experiments with n = 23 for emulsion gel and Aldara and n = 17 for untreated control. *Significant difference with p<0.05 by Mantel Cox test compared to the untreated control group.

In the Aldara-based TCI group, 21 out of 23 animals responded to the treatment, as shown by a reduction in tumor size. However, we observed a tumor relapse in seven mice, leaving in a durable protection in 14 of 23 mice (overall survival 60.8%, median survival not reached) (Fig. 5B). In contrast, all animals treated with IMI-Gel-based TCI initially responded to vaccination treatment with decreasing tumor sizes (Fig. 5C). However, the tumors relapsed in six mice, leading to an overall survival of 73.9% (median survival not reached, Fig. 5D). While there was a trend for higher survival for IMI-Gel-treated mice compared the Aldara group, this did not reach statistical significance (p = 0.07 by Mantel-Cox test).

In summary, our results suggest that the vaccination potency of IMI-Gel-based TCI is at least as effective as Aldara-based TCI in the induction of tumor specific immunity despite lower imiquimod permeation through the skin.

## Discussion

Although standard vaccination approaches are effective in a considerable number of infectious diseases [19], vaccination strategies against tumors have only recently begun to prove successful [20]. Despite the limited efficacy of Sipuleucel-T, the FDA has recently approved this DC vaccine for the treatment of advanced prostate cancer, further underlining the medical need for therapeutic cancer vaccines [21]. Moreover, peptide-based cancer vaccine approaches are effective, e. g. in renal cancer with GM-CSF as adjuvant [22]. While classical prophylactic vaccination approaches are suitable for inducing protective antibody responses against virus infections, they may not be ideal for the induction of therapeutic T-cell responses. In this context, transcutaneous vaccination approaches may be an attractive way to deliver antigens and adjuvants. The proof-of-concept has been demonstrated already years ago [6], [8], [10]. We have been following a TCI approach based on a CTL epitope and the TLR7 agonist imiquimod formulated in Aldara. While we observed primary CTL responses [8], [11] and anti-tumor effects of Aldara-based TCI [5], [9], this particular TCI method is limited by inefficient memory CTL generation. Aldara-based TCI efficiency can be increased by costimulatory signals like CD40 ligation [9] or UV-B irradiation [5] leading to enhanced memory formation and improved tumor protection. An important limitation of our transcutaneous vaccination approach concerns the use of a mouse model, which on the one hand allows the evaluation of this novel treatment approach in a preclinical animal model. On the other hand, the usage of mouse models does not account for differences between human and mouse skin, in the latter the stratum corneum being significantly thinner and better permeable for transcutaneous drug delivery [23]. In addition, differences of murine and human APCs in TLR responsiveness or antigen presentation need to be taken into account [1], [24] and limit applicability and the direct translation of our results to the application in humans. On the other hand, the topical application of imiquimod has proven efficacy for the treatment of patients with HPV infections [12] and skin cancers [13] as well as when used as an adjuvant for vaccination [14], [15] suggesting that this approach may be also feasible and effective in humans.

Based on our previous observation that imiquimod with peptide also induces CTL responses independent of complete solubilisation (as in Aldara) [16], we manufactured the novel imiquimod formulation IMI-Gel in which imiquimod is nano-dispersed in a hydrophilic polyacrylate gel. We now characterized IMI-Gel physicochemical properties as stable over at least nine months at room temperature. This compares favourably with imiquimod in Aldara, which is delivered in sachets for single use, increasing the manufacturing expenses. Moreover, the IMI-Gel formulation on the basis of a hydrophilic gel now allows for the addition of hydrophilic components, such as other adjuvants or peptide antigens which has been a major limitation of a TCI approach using Aldara. Not surprisingly, both crystalline imiquimod and the gel formulation show a lower skin-permeation rate compared to Aldara which results in a greater amount of imiquimod recovered from the skin surface and an approx. 10fold decreased drug permeation across mouse skin (Fig. 2). However, we detected comparable amounts of imiquimod within the skin, which is in support of the notion that this is the place where the drug is needed for DC activation. Currently, we do not know in detail how the particle size of imiquimod crystals in IMI-Gel affects the TCI induced immune response although this is suggestive based on the work of others [25]. However, a decreased systemic drug exposure should not adversely affect vaccination efficacy since local interaction of the immunostimulator imiquimod with APCs in the epidermis and dermis should potentially be most important [5], [10]. Our demonstration that imiquimod formulated in Aldara and IMI-Gel formulations induce CTL responses with equal efficacy (Fig. 3) supports this hypothesis. In contrast to parenteral vaccine delivery methods, the transcutaneous route directly accesses relevant skin-resident APC populations [5], [10] while the s. c. injection or oral application of IMI-Gel and peptide fails to induce a CTL response (Fig. 4).

Remarkably, when directly comparing IMI-Gel-based TCI to Aldara-based TCI in a therapeutic tumor rejection assay, we observed that all mice in the IMI-Gel group responded to the treatment with a decrease in tumor size and a lower number of animals relapsed, leading to an improved overall survival. Given the number of animals in the experimental groups, the differences were not statistically significant (p = 0.07 by Mantel-Cox test, comparing IMI-Gel vs. Aldara). From our previous work, we know that Aldara-based TCI is not an ideal tumor vaccine since anti-tumor responses can be significantly augmented by additional stimulation such as UV exposure or CD40 triggering [5], [9]. This is an obvious limitation of these tumor rejection assays. Nevertheless, our results allow the conclusion that our novel imiquimod formulation IMI-Gel is a suitable and feasible basis for the further development in terms of enhancing vaccination efficacy, e. g. by combination with other TLR agonists [26] or CD40 triggering [9]. We also observed tumor rejections in the non-vaccinated control group, accompanied by specific CTL responses only in the animals that rejected the tumors. This is in contrast to our previous experiments [5],[9], in which we had not observed any spontaneous tumor rejections. The occurrence of such immune responses in the current experiments can only be explained by the induction of CTL at the time of tumor inoculation, potentially due to a significant number of necrotic cells in the E.G7 inoculations [27]. Spontaneous tumor rejections should not compromise the validity of the experimental system since (i) it can be assumed that they occurred equally over all experimental groups and (ii) CTL responses were absent in tumor-bearing mice. Therefore, it is safe to conclude that TCI with IMI-Gel is at least as effective as TCI with Aldara despite the 10fold lower skin permeation of imiquimod.

Taken together, we developed a novel imiquimod-based formulation with interesting pharmaceutical and immunological properties that should be used for the development of TCI approaches. A deeper understanding of the underlying mechanisms may harbour the key for a next-generation vaccination platform that can be used for the treatment of persistent infections and cancer.

## Materials and Methods

### Ethics Statement

All animal studies were conducted according to the national guidelines and were reviewed and confirmed by an institutional review board/ethics committee headed by the local animal welfare officer (Prof. Dr. O. Kempski) of the University Medical Center (Mainz, Germany). The National Investigation Office Rheinland-Pfalz (Koblenz, Germany) finally approved the animal experiments (AZ 23 177-07/G11-1-034 and 23 177-07/G13-1-012).

### Materials

Imiquimod and Azone were obtained from Chemos GmbH (Regenstauf, Germany). Jojoba wax, polysorbate 80, polyacrylic acid, sodium hydroxide, sodium acetate trihydrate, and glacial acetic acid were supplied by Carl Roth GmbH (Karlsruhe, Germany). Trifluoric acid was provided by Sigma-Aldrich (Steinheim, Germany). Acetonitrile and ethanol, both HPLC grade, were obtained from VWR (Darmstadt, Germany). Officinal cremor basalis according to DAC was obtained from Caesar and Loretz GmbH (Hilden, Germany).

### Production of IMI-Gel

For pre-homogenization, imiquimod was added to a 9 mg/ml aqueous solution of polysorbate 80 in a grinding vessel. Milling was performed for six cycles to ensure an appropriate pre-homogenization as well as a particle size below 30 µm to establish a safe and reliable function during the subsequent high-pressure homogenization (HPH) process.

After sieving, polysorbate 80 was added again to ensure a stable emulsion. Moreover, Azone and jojoba wax were added (2.5% and 42.5%, w/w, respectively). HPH was performed by an Emulsiflex C3 (Avestin) for five cycles at 500 bar and ten cycles at 1000 bar, respectively. The resulting oil in water emulsion with suspended imiquimod nanoparticles appeared as a yellow fluid. In order to create a semisolid formulation, a previously prepared and precisely neutralized polyacrylic acid gel was added. Additionally, we investigated whether a storage period of nine months under room conditions affects imiquimod particle size and dispersity under measurement settings described below.

### Electron micrographs

Samples were spread on a glass slide and then adsorbed onto a continuous carbon grid. They were washed three times with 20 µl H_2_O distilled prior to staining with 5 µl of a 1% uranyl acetate solution. After the staining solution was blotted off, grids were air-dried. They were transferred to an electron microscope and images were recorded using a 4 k×4 k TemCam-F416 (TVIPS, Munich, Germany).

### Rheologic studies

Rheograms were obtained and analyzed as described previously [16] using a Haake Rheostress 1 viscosimeter with a cone and plate device PiT-L 35 and RheoWin 4 data manager software. Flow curves display shear stress vs. shear rate and were obtained at a predefined shear rate of 0–200 s^−1^, recording the resulting shear stress. Thixotropy was determined by a controlled shear rate with a rate of 0–1000 s^−1^ for 60 s, following a 1000 s^−1^ phase for 30 s and subsequent reduction of the shear rate from 1000 to 0 s^−1^ for a further 60 s. The experiments were performed at 23.0°C.

### Particle size determination

Visualization of imiquimod particles embedded in the emulsion gel matrix (IMI-Gel) was performed by electron microscopy. To determine particle sizes within the formulation, dynamic light scattering (DLS) measurements were performed using a Zeta Sizer nano (Malvern Instruments GmbH, Herrenberg, Germany). Briefly, 50 µl of IMI-Gel was diluted with 4 ml double distilled water. Then, 100 µl of the resulting suspension was additionally diluted with 1.3 ml of double distilled water in a disposable cuvette. Measurements were performed directly after the manufacturing process or nine months post manufacturing to assess the occurrence of Ostwald-ripening. Each sample was prepared three times. Z-average values were measured by Zeta Sizer nano. Then, particle sizes were calculated as the mean value of three z-average measurements. In order to give an overview of particle size range, martin diameter of 25crystals from the electron microscopic specimen was determined by open source ImageJ software.

### Permeation assays

Male or female C57BL/6 mice at 6–8 weeks were obtained from the local animal facility of the University of Mainz. The animals were sacrificed and dorsal hair was removed with electric clippers. Skin samples were prepared and fat was removed using a scalpel. Skin (0.79 cm^2^) was treated with either 50 mg Aldara or IMI-Gel, both containing 5% imiquimod. Afterwards skin samples were placed in an EDC-07 Franz-diffusion-cell model (Labswiss, Muttenz, Switzerland). The acceptor chamber contained a blend of sodium acetate trihydrate/glacial acetic acid buffer (20 µM) and ethanol (7/3 v/v) with a resulting pH of 3.6, previously degassed by an ultra sound bath for appropriate duration. Temperature was set at 32°C and a magnetic stirrer constantly agitated acceptor media. Samples were collected after 1, 2, 3, 5, 7, 8.5 and 24 hours. To quantify imiquimod concentrations, a 300 C8 5 µm reversed phase RP 250*4.6 mm column (Mainz Analysentechnik, Mainz, Germany) was used. Mobile phase comprises double distilled water, trifluoric acid and acetonitril (70∶0.0125∶30 V/V). This mobile phase provided a pH value of 2.8 to avoid imiquimod precipitation in the column. Flow rate was 1.0 ml/min ensured by a Jasco PU-980 Intelligent HPLC pump (JASCO Germany GmbH, Gross-Umstadt, Germany). For quantitative API detection UV absorbance was determined by a UV detector (JASCO Germany GmbH, Groβ-Umstadt, Germany) at 245 nm wavelength. Imiquimod eluted after 5.5 minutes. Detectable concentration ranges was from 35–1790 ng/ml. Jasco-Borwin HSS-2000 software was used to analyze revealed peaks.

### Quantification of imiquimod in the skin

Mice were treated with either 50 mg Aldara or IMI-Gel on the shaved dorsum (6 cm^2^). Quantification of imiquimod from skin samples and skin surface was performed after 3 hours using reversed phase HPLC, using a modified method similar to De Paula et al. [28].

Briefly, skin (1 cm^2^) was homogenized and extracted with 3 ml extraction buffer (7∶3 (v/v) MeOH:acetate buffer (pH 4.0, 100 mM).

To determine residual imiquimod on the skin surface, skin was wiped thoroughly with gauze and the gauze pad extracted with 3 ml of extraction buffer.

HPLC was performed using a Dionex Ultimate 3000 HPLC equipped with a UV-Vis detector. Detection wavelength was 242 nm. Buffer A was 100 mM Acetate Buffer pH4.0 Buffer B was 100% Acetonitrile. Samples were analysed on a 2 mm×50 mm Phenomenex Max RP (C-12) column using a gradient from 5% B to 80% B in 7 min.

Column was reequilibrated to starting conditions for 5 min. The flow rate was 250 µl/min. Column compartment was thermostatted at 50°C. Under these experimental conditions, imiquimod eluted at 5.25 min. Total run time was 12 min and the injection volume was 5 µl.

### Transcutaneous immunizations

Transcutaneous immunizations were described previously [5]. Briefly, dorsal hair was removed with electric clippers. For TCI, mice were anesthetized by i. p. injection with ketamine (Ratiopharm, Ulm, Germany; 71.2 mg per mouse) and Rompun 2% (Bayer Health Care, Leverkusen, Germany;0.2 mg per mouse). 50 mg Aldara containing 5% imiquimod (Meda Pharma, Wangen-Brüttisellen, Switzerland) together with peptide (OVA_257–264_, SIINFEKL, 100 µg in DMSO, provided by S. Stevanovic, Department of Immunology, Institute for Cell Biology, University of Tübingen, Germany) were applied on the shaved dorsum (approx. 3 cm×5 cm) on days 0 and 1. Alternatively mice were treated with 50 mg of IMI-Gel also containing 5% imiquimod followed by application of officinal cremor basalis together with 100 µg SIINFEKL.

For immunizations s. c. IMI-Gel (100 mg per mouse) was diluted in 80 µl distilled water. After adding 200 µg SIINFEKL peptide, the solution was injected in the dorsal neck region of mice on day 1.

For oral immunization, IMI-Gel (50 mg per mouse) was diluted with 40 µl distilled water and 100 µg SIINFEKL peptide. Mice were fed on days 0 and 1.

### Tumor rejection assay

Tumors were inoculated by s. c. injection of E.G7 thymoma cells (4×10^5^, from ATCC) as described previously [5]. Tumors were allowed to grow until palpable before treatments started. Mice were immunized in weekly intervals over a period of three weeks. Tumor size was monitored every other or third day at least three times per week with a caliper in two dimensions. During the observation times the mice had no indication of discomfort as indicated by lethargy or piloerection. To further avoid animal suffering, mice were sacrificed when tumor size exceeded 20 mm in length and width by CO_2_ asphyxiation. The day subsequent to euthanasia was defined as the day of death.

### Flow cytometric analyses and *in vivo* cytotoxicity assay

The following mAbs were used for flow cytometric analyses: Pacific Blue-conjugated anti-CD8 (clone 53–6.7), APC-conjugated anti-CD44 (clone IM7) and FITC-conjugated anti-CD62L (clone MEL-14), all from eBioscience, Frankfurt, Germany. Blood samples were collected after tail vein incision. After a hypotonic lysis step samples were incubated with mAbs on ice. H2-K^b^-SIINFEKL-specific T cells were detected by H2-K^b^ tetramer staining as described previously [11]. *In vivo* cytolytic activity was assessed by transfer of 2×10^7^ target cells labelled with either 4 µM (CFSE^high^) or 0.4 µM (CFSE^low^) carboxyfluorescein diacetate succinimidyl ester. The CFSE^low^ cells were additionally loaded with SIINFEKL (2 µM). Both populations were transferred i.v. in 1∶1 ratio. Splenocytes of immunized and control mice were analysed by flow cytometry. All analyses were performed with a LSRII Flow Cytometer and FACSDiva software (BD Pharmingen, Hamburg, Germany).

### Statistical analysis

All statistical analyses were performed using GraphPad Prism (version 5.0a for Mac OS X, GraphPad Software, San Diego California USA, www.graphpad.com). Survival analyses were performed by the Mantel-Cox test. For comparison between two groups a two-tailed Student’s *t* test was used. Comparisons of multiple groups were performed by one-way ANOVA with Bonferroni’s posttest. For all analyses, p<0.05 was considered as statistically significant.
